This article has been retracted.

# miR-96-5p enhances cell proliferation and invasion via targeted regulation of ZDHHC5 in gastric cancer

**DOI:** 10.1042/BSR20191845

**Published:** 2020-04-15

**Authors:** Baolong Wang, Xianrong Liu, Xiangtao Meng

**Affiliations:** 1 General Surgery, ShanXian Hygeia Hospital, Heze, Shandong Province, China; 2 Outpatient Department, ShanXian Central Hospital, Heze, Shandong Province, China; 3 General Surgery, DongDa Hospital of ShanXian, Heze, Shandong Province, China

**Keywords:** cell apoptosis, gastric adenocarcinoma, microRNA-96-5p, prognosis

## Abstract

**Objective:** To explore the biological function and mechanism of miR-96-5p in gastric cancer.

**Methods:** The expression of differently expressed microRNAs (DEMs) related to gastric adenocarcinoma (GAC) prognosis was identified in GAC tumor samples and adjacent normal samples by qRT-PCR. A target gene miR-96-5p was selected using TargetScan, miRTarBase, miRDB databases. The combination of miR-96-5p and ZDHHC5 was verified by luciferase receptor assay. To further study the function and mechanism of miR-96-5p, we treated MGC-803 cells with miR-96-5p inhibitor and si-ZDHHC5, then detected cell viability, apoptosis, migration and invasion ability, as well as the expression of ZDHHC5, Bcl-2, Bax, cleaved caspase-3, cleaved caspase-9, and COX-2 by Western blot.

**Results:** Compared with adjacent normal samples, the levels of miR-96-5p, miR-222-5p, and miR-652-5p were remarkably increased, while miR-125-5p, miR-145-3p, and miR-379-3p were significantly reduced in GAC tumor samples (*P*<0.01), which were consistent with bioinformatics analysis. Furthermore, ZDHHC5 was defined as a direct target gene of miR-96-5p. miR-96-5p silence significantly reduced cell viability, increased cell apoptosis, and suppressed cell migration and invasion, as well as inhibited the expression of Bcl-2 and COX-2 and promoted Bax, cleaved caspase-3 and cleaved caspase-9 level in MGC-803 cells (*P*<0.01). Notably, ZDHHC5 silence reversed the inhibiting effects of miR-96-5p on MGC-803 cells growth and metastasis

**Conclusion:** Our findings identified six microRNAs (miRNAs; miR-96-5p, miR-222-5p, miR-652-5p, miR-125-5p, miR-145-3p, and miR-379-3p) related to GAC prognosis, and suggested that down-regulated miR-96-5p might inhibit tumor cell growth and metastasis via increasing ZDHHC5 expression enhance MGC-803 cell apoptosis, as well as decrease MGC-803 cell metastasis.

## Introduction

Gastric adenocarcinoma (GAC) is the most common malignant tumor originating in the stomach, with approximately 951000 diagnosed cases and 723000 deaths in 2012 [1,2]. At present, the common and effective treatment method is to combine surgery with adjuvant radiotherapy or chemotherapy to improve the 5-year survival rate of GAC [3]. However, due to atypical symptoms of early GAC, most patients with proximal or distal metastases find delayed diagnosis, which leads to poor treatment and prognosis [4]. Thus, it is essential to reveal novel diagnostic and therapeutic targets for GAC.

It is well known that a major challenge of GAC treatment is poor prognosis, and environmental exposures and genetic mutations have been identified to be associated with this outcome [5]. A large body of evidence indicates that the poor prognosis of GAC is significantly associated with many molecular biomarkers such as microRNA (miRNA) [6,7]. miRNAs, as endogenous non-coding small-molecule RNAs, widely exist in severe conditions [8]. It has been revealed that a large number of miRNAs are involved in various biological functions such as cell differentiation, apoptosis, migration, invasion, and proliferation in human diseases through post-transcriptional regulation of gene expression [8,9]. Previous studies have demonstrated that miRNA disorders can significantly influence the prognosis of patients with gastric cancer, such as miR-203 [10], miR-21 [11], and miR-25 [12]. Imaoka et al. [10] have reported that a low serum miR-203 expression is related to poor prognosis, and which is considered as a noninvasive biomarker for prognosis of gastric cancer patients. Simonian et al. [11] also have evidence that circulating miR-21 can be considered as a diagnostic and prognostic biomarker for gastric cancer. In addition, Li et al. [12] revealed that miR-25 is associated with the prognosis of gastric cancer, and can induce cell migration and proliferation by targeting transducer of ERBB2, 1. Therefore, it is important to find novel miRNAs related to the prognosis of GAC that may contribute to the development of GAC diagnosis.

In the current study, the miRNA expression data of GAC based on The Cancer Genome Atlas (TCGA) were analyzed to screen differently expressed miRNAs (DEMs) and DEMs related to GAC prognosis. In addition, DEMs were identified in clinical samples and the mechanism of DEM was investigated *in vitro*. Based on this, we aimed to search for new therapeutic targets for GAC, and provide some useful insights in improving the prognosis of GAC patients.

## Materials and methods

### Data extraction and DEMs screening

Based on the Illumina HiSeq 2000 RNA Sequencing Platform platform, miRNA expression profile data (level 3) and corresponding GAC clinical information were downloaded from TCGA (https://portal.gdc.cancer.gov/). A total of 452 samples were obtained from this dataset, including 410 GAC tumor samples and 42 normal control samples. The edgeR package in R was utilized to screen DEMs between GAC samples and normal samples. The thresholds were defined as false discovery rate (FDR) < 0.05 and |log fold change (FC)| > 1. Meanwhile, volcano plots and heat maps were generated based on the obtained DEMs.

### DEMs screening related to prognosis

The overall survival (OS) time was individually extracted from clinical information. Then, combined with the OS times and the expression levels of DEMs, DEMs related to prognosis were screened using KMsurv package of R, with the threshold of log-rank *P*<0.05.

### Clinical validation sample collection

The present study obtained ethical approval from the ethics committee of DongDa Hospital of ShanXian, and the study was performed according to the Helsinki Declaration. Twenty paired adjacent normal tissues and GAC tumor tissues were collected from October 2017 to October 2018 in our hospital. All samples were confirmed by HE staining and stored in RNA later. Meanwhile, peripheral blood from these GAC patients and 20 paired healthy subjects were obtained. The clinical information, including age, weight, gender, distant metastasis, lymph node metastasis, depth of invasion, and TNM stage are shown in Table 1.

**Table 1:** Distribution of characteristics in GAC patients and healthy subjects

Variables	Patients (*n*=20)		Controls (*n*=20)		*P*^1^
	*n*	%	*n*	%	
Age (years, mean ± SD)	62.1 ± 5.2		60.1 ± 10.2		0.73
Weight (kg, mean ± SD)	64.0 ± 7.1		69.1 ± 6.6		0.88
Gender					
Male	13	65.0	1	55.0	0.64
Female	7	35.0	9	45.0	
Depth of invasion					
T1/T2	7	35.0	-	-	-
T3/T4	13	65.0	-	-	-
Lymph node metastasis					
N0	6	30.0	-	-	-
N1/N2/N3					
	14	70.0			
Distant metastasis					
M0	8	40.0	-	-	-
M1	12	60.0	-	-	-
TNM stage					
I/II	7	35.0	-	-	-
III/IV	13	65.0	-	-	-

1 Independent-samples *t* test and two-sided χ^2^ test for selected variables distributions between cases and controls.

### Predicting target genes of DEMs

Target genes of DEMs related to prognosis were predicted using the three online analysis databases, including miRDB, miRTarBase, and TargetScan. Overlapping target genes among the three tools were selected to make the bioinformatics analysis more reliable. Then, the Venn diagram online tool was used to obtain the intersection of predicted target genes between the three databases, and the target genes that overlapped in the three databases were considered as potential target genes for DEM.

### Cell culture and transfection

Human gastric carcinoma cell line MGC-803 was obtained from Shanghai Obio Technology Co., Ltd. The cells were maintained in Dulbecco’s Modified Eagle’s Medium (DMEM, Gibco, Carlsbad, CA, U.S.A.) supplemented with 10% fetal bovine serum (FBS, Gibco, Carlsbad, CA, U.S.A.). MiR-96-5p mimics, mimic negative control (NC), miR-96-5p inhibitor, inhibitor NC, ZDHHC5 silence vector (si-ZDHHC5), and si-NC were constructed by Biosyntech Co., Ltd (Suzhou, China). MGC-803 cells were inoculated in six-well plates for 24 h with approximately 5 × 10^5^ cells in each well, and then the above vectors were transfected into MGC-803 cells by Lipofectamine 2000 (Invitrogen, Carlsbad, CA, U.S.A.) according to manufacturer’s instructions. Meanwhile, MGC-803 cells without transfection served as control group.

### Real-time quantitative polymerase chain reaction

Total RNA from tissues and peripheral blood was obtained by TRIzol (Invitrogen) and RNeasy Plus Mini Kit (Qiagen, Valencia, California, U.S.A.) according to the manufacturer’s instructions. The concentration of RNA was detected using NanoDrop ND-2000 (Invitrogen). Mir-X™ miRNA FirstStrand Synthesis Kit (Takara, Dalian, China) was used utilized to obtain cDNA by reverse transcription of RNA. The quantitative polymerase chain reaction (qPCR) was carried out using the SYBR Premix Ex Taq™ II (Takara) by ABI 7900 qRT-PCR System (Applied Biosystems, Foster City, CA, U.S.A.). The primers sequences are listed in Table 2. U6 was used as the internal control for measuring miRNA level, and GAPDH was served as the internal control of for measuring ZDHHC5 expression. Data were analyzed with 2^−ΔΔ*C*_t_^ method.

**Table 2:** Primers used for the qRT-PCR related sequence

Gene	Primer sequence
*miR-96-5p*	F: 5′-TCAACTGGTGTCGTGGAGTCGGCAATTCAGTTGAGAGCAAAAA-3′
	R: 5′-ACACTCCAGCTGGGTTTGGCACTAGCACATT-3′
*miR-125a-5p*	F: 5′-CCCTGAGACCCTTTAACCT-3′
	R: 5′-GTCCAGTTTTTTTTTTTTTTTCACAG-3′
*miR-145-3p*	F: 5′-GGTCCAGTTTTCCCAGGA-3′
	R: 5′-CCAGTTTTTTTTTTTTTTTAGGGATTC-3′
*miR-222-5p*	F: 5′-GCTCAGTAGCCAGTGTAGA-3′
	R: 5′-GTCCAGTTTTTTTTTTTTTTTAGGATCT-3′
*miR-379-3p*	F: 5′-GCAGTGGTAGACTATGGAAC-3′
	R: 5′-GGTCCAGTTTTTTTTTTTTTTTCCT-3′
*miR-652-5p*	F: 5′-CCTAGGAGAGGGTGCCA-3′
	R: 5′-GTCCAGTTTTTTTTTTTTTTTGAATGG-3′
*miR-708-3p*	F: 5′-GCAACTAGACTGTGAGCTTC-3′
	R: 5′-GGTCCAGTTTTTTTTTTTTTTTCTAGA-3′
*ZDHHC5*	F: 5′- GAAGACTGAAGAAAGATAAGAGACATTG-3′
	R: 5′-GACACTTCAAAAGTTTACTGTGGATG-3′
*GAPDH*	F: 5′-AGAAGGCTGGGGCTCATTTG-3′
	R: 5′-AGGGGCCATCCACAGTCTTC-3′
*U6*	F: 5′-AGGGGCCATCCACAGTCTTC-3′
	R: 5′-AACGCTTCACGAATTTGCGT-3′

### Luciferase reporter assay

The target gene of miR-96-5p was verified using the luciferase reporter assay. The 3′-UTR-wild-type (WT) or mutant (MUT) of ZDHHC5 was cloned into a pGL3-basic vector, named as ZDHHC5-WT and ZDHHC5-MUT. Then, ZDHHC5-WT or ZDHHC5-MUT and phRL-TK plasmid were co-transfected with miR-96-5p mimic or miR-96-5p NC (synthesized by Biosyntech, Suzhou, China) into 293T cells, respectively, for 48 h using Lipofectamine 2000. Finally, the measurement of the relative luciferase activities was carried out by the Dual-Glo Luciferase Assay System (Promega) as per the manufacturer’s introductions.

### Cell viability assay

MGC-803 cells were subjected to various transfections and then grown in 96-well plates. After conventional incubation for 24, 48, 72, and 96 h, each well was added with 10 μl of MTT (5 mg/ml, Sigma) for another 4 h. Afterward, 100 μl of dimethyl sulfoxide was added. Microplate spectrophotometer was used to evaluate cell viability based on the absorbances at 470 nm.

### Cell apoptosis assay

FITC-Annexin V Apoptosis kit was used in this experiment. Trypsin was used to digest cells with various treatments, and then cells were harvested. Next, cells were rinsed with PBS, and resuspended with Binding Buffer. After the incubation of FITC-Annexin V and PI with cells for 15 min, flow cytometer (BD, CA, U.S.A.) was used to calculate the number of apoptotic cells.

### Transwell assay

Tumor cell invasion and migration were elevated by Transwell chambers (Corning). Concretely, the bottom compartment was added with DMEM with 10% FBS. The transfected cells were grown in the upper compartment coated with Matrigel Matrix and cultured in medium free of serum for 24 h. Subsequently, the cells in the bottom compartment was fixed and stained with 4,6-diamidino-2-phenylindole. An inverted microscope (Olympus, Japan) was utilized to evaluate cell migration and invasion.

### Western blotting

Total proteins were isolated by RIPA Lysis Buffer (Beyotime, Shanghai, China). Proteins’ concentrations were tested by bicinchoninic acid (BCA) kit (Beyotime). The protein sample was separated on SDS/PAGE gel, and transferred to polyvinylidene fluoride membranes, followed by the blockage with 5% nonfat milk for 1 h. Next, the membranes were probed with primary antibodies of ZDHHC5 (1:1000, Proteintech), Bcl-2 (1:1000, Abcam), Bax (1:1000, Abcam), pro-caspase-3 (1:1000, Abcam), cleaved-caspase-3 (1:1000, Abcam), pro-caspase-9 (1:1000, Abcam), cleaved-caspase-9 (1:1000, Abcam), COX-2 (1:1000, Abcam), and GAPDH (1:1000, Beyotime) overnight at 4°C. Then, membranes were incubated with secondary antibody (1:1000, Beyotime) for 2 h keeping in a dark place at room temperature. The protein levels were detected by enhanced chemiluminescence (ECL) Plus reagent (Beyotime).

### Statistical analysis

Statistical analysis was conducted using SPSS Statistics software 22.0 (Chicago, IL, U.S.A.). Continuous variables were expressed as mean ± standard derivation (SD) and analyzed by independent-samples *t* test. Categorical variables were expressed as percentages and assessed by two-sided chi-square test. The differences of multiple groups were performed by one-way ANOVA following with post-hoc Dunnett *t* test. *P*<0.05 was considered to be statistically significant.

## Results

### DEMs between GAC sample and normal sample based on TCGA

According to the selective criteria, a total of 299 DEMs were identified between GAC and normal control samples, including 225 up-regulated and 74 down-regulated miRNAs. As shown in Figure 1A,B, volcano plots and heat maps were conducted for these 299 DEMs.

**Figure 1:** DEMs between GAC sample and normal sample (**A**) Volcano plots for DEMs expression. Dark dots represent up-regulated miRNAs, whereas lighter dots represent down-regulated miRNAs. (**B**) Hierarchical gene clustering analysis of DEMs showed by heat map. Dark represents up-regulated miRNAs, whereas lighter represents down-regulated miRNAs.

### DEMs related to prognosis based on TCGA

Based on these 299 DEMs, the relationship between patient OS and miRNA expression was evaluated, and the results showed that 35 DEMs were significantly related to the prognosis of GAC patients (*P*<0.05). Among these DEMs, there are seven miRNAs that have a higher correlation with GAC prognosis (*P*<0.01), including miR-96-5p (*P*=8.049 × 10^−3^), miR-125-5p (*P*=9.638 × 10^−4^), miR-145-3p (*P*=6.002 × 10^−3^), miR-222-5p (*P*=1.812 × 10^−3^), miR-379-3p (*P*=5.032 × 10^−3^), miR-652-5p (*P*=3.145 × 10^−3^), and miR-708-3p (*P*=7.984 × 10^−3^) (Figure 2).

**Figure 2:** Association of DEMs with OS of GAC Dark lines represent high expression and lighter lines represent low expression.

### DEMs identification in clinical samples

A total of 20 GAC patients and 20 healthy subjects were included in the present study. There were no significant differences in age, weight, and gender between GAC patients and healthy subjects (Table 1). Based on the above survival analysis, six miRNAs were selected to identify in GAC tumor samples and adjacent normal samples. RT-qPCR showed that compared with adjacent normal samples, the levels of miR-96-5p, miR-222-5p, and miR-652-5p were remarkably increased, while miR-125-5p, miR-145-3p, and miR-379-3p levels were obviously reduced in GAC tumor samples (*P*<0.01, Figure 3A), which was consistent with bioinformatics analysis results by TCGA. Moreover, miR-96-5p levels were detected in the blood of GAC patients and healthy subjects, while no significant differences were found (Figure 3B).

**Figure 3:** The identification of DEMs levels in GAC patients and healthy subjects (**A**) The levels of miR-96-5p, miR-222-5p, miR-652-5p, miR-125-5p, miR-145-3p, and miR-379-3p in tumor sample and adjacent normal samples by RT-qPCR. (**B**) The miR-96-5p level in blood of GAC patients and healthy subjects by RT-qPCR. (**) denotes difference from control (*P*<0.05). Values are means ± SD.

### Target gene prediction and identification of miR-96-5p

Considering that miR-96-5p has the highest correlation with GAC prognosis, the function of miR-96-5p was investigated in the following experiments. It was found that a total of 39 overlapping target genes existed in the TargetScan, miRTarBase, and miRDB databases (Figure 4A). Based on this bioinformatics analysis, *ZDHHC5* was considered as a potential target gene of miR-96-5p (Figure 4B). Luciferase receptor assay showed that after co-transfection with ZDHHC5-WT and miR-96-5p mimic, the relative luciferase activity was reduced compared with co-transfection with miR-96-5p NC, while significant difference was not found after ZDHHC5-MUT treatment (Figure 4C), which suggested ZDHHC5 as a direct target gene of miR-96-5p. In addition, the mRNA level of ZDHHC5 was obviously decreased in cells with miR-96-5p mimic, and remarkably increased after transfection with miR-96-5p inhibitor (*P*<0.01, Figure 4D).

**Figure 4:** Target gene prediction and identification of miR-96-5p (**A**) The intersection of the predicting target genes of miR-96-5p among the TargetScan, miRTarBase, and miRDB databases using Venn diagram. (**B**) Prediction of the binding site of miR-96-5p to ZDHHC5 by bioinformatics. (**C**) Target regulation of miR-96-5p to ZDHHC5 proved by luciferase reporter system. (**D**) The mRNA level of ZDHHC5 in MGC-803 cells transfected with miR-96-5p mimic, miR-96-5p inhibitor or their corresponding control by qRT-PCR.

### Effect of miR-96-5p on tumor growth and metastasis through ZDHHC5 in MGC-803 cells

To further study the effect of miR-96-5p on GAC, the miR-96-5p inhibitor was used to silence miR-96-5p level in MGC-803 cells. It was found that the mRNA level of ZDHHC5 was obviously down-regulated after transfection with si-ZDHHC5 compared with si-NC in MGC-803 cells (*P*<0.01, Figure 5A). Moreover, miR-96-5p silence prominently inhibited cell viability (*P*<0.05, Figure 5B), promoted cell apoptosis (*P*>0.05, Figure 5C), and decreased cell migration and invasion (*P*<0.01, Figure 5D,E). Notably, co-transfection of miR-96-5p inhibitor and si-ZDHHC5 exerted the opposite effects in comparison with miR-96-5p inhibitor treatment (Figure 5B–E). In addition, the expression of apoptosis-related proteins (Bcl-2, Bax, cleaved caspase-3, cleaved caspase-9, and COX) was detected by Western blot. The results revealed that compared with MGC-803 cells without treatment, miR-96-5p silence inhibited the expression of Bcl-2 and COX-2, as well as increased the expression of Bax, cleaved caspase-3, and cleaved caspase-9 (apoptosis proteins) in MGC-803 cells (*P*<0.01, Figure 5F), while the expression of these proteins revealed a opposite trend after co-transfection of miR-96-5p inhibitor and si-ZDHHC5 (*P*<0.01, Figure 5F).

**Figure 5:** miR-96-5p silence inhibits tumor growth and metastasis in MGC-803 cells (**A**) The mRNA level of ZDHHC5 in MGC-803 cells transfected with si-NC, si-ZDHHC5 by qRT-PCR. (**B**) Cell viability in MGC-803 cells transfected with miR-96-5p inhibitor, miR-96-5p inhibitor + si-ZDHHC5, or their corresponding controls by MTT assay. (**C**) The rate of apoptotic cells in MGC-803 cells transfected with miR-96-5p inhibitor, miR-96-5p inhibitor + si-ZDHHC5, or their corresponding controls by flow cytometry analysis. (**D,E**) Cell migration and invasion in MGC-803 cells transfected with miR-96-5p inhibitor, miR-96-5p inhibitor + si-ZDHHC5, or their corresponding controls by Transwell assay. (**F**) The protein levels of COX-2, Bcl-2, Bax, pro-caspase-3, cleaved-caspase-3, pro-caspase-9, and cleaved-caspase-9 in MGC-803 cells transfected with miR-96-5p inhibitor, miR-96-5p inhibitor + si-ZDHHC5, or their corresponding controls by Western blotting. (*) denotes difference from control (P<0.01); (**) denotes (*P*<0.05); (***) denotes (*P*>0.05). Values are means ± SD.

## Discussion

In the present study, based on miRNA expression profile data from TCGA, a total of 299 DEMs and 35 DEMs related to the prognosis of GAC were screened. Then, six miRNAs were selected to identify in GAC tumor samples and adjacent normal samples, and the results were consistent with bioinformatics analysis. In addition, miR-96-5p is considered an important biomarker and has been studied in the following *in vitro* experiments. Our results revealed that ZDHHC5 was a direct target gene of miR-96-5p, and miR-96-5p silence reduced cell viability, increased cell apoptosis, and suppressed cell migration and invasion in MGC-803 cells, while ZDHHC5 silence partly reversed the effects of miR-miR-96-5p down-regulation on tumor cell growth and metastasis.

Six miRNAs were identified in the present study, and the results showed that the levels of miR-96-5p, miR-222-5p, and miR-652-5p were overexpressed, while miR-125-5p, miR-145-3p, and miR-379-3p levels were down-regulated in GAC sample. Several studies have demonstrated that miR-96-5p is overexpressed in various cancers, including colorectal cancer [13], pancreatic carcinoma [14], prostate cancer [15], hepatocellular carcinoma [16], and breast cancer [17], and it is oncogene that promotes cell proliferation. It has been reported that miR-652-5p is associated with non-small cell lung cancer [18], esophageal adenocarcinoma [19], and breast cancer [20], while the mechanism of miR-652-5p was not elaborated. Current research on miR-222-5p has focused on the role of angiogenesis in the endothelium [21,22], and few studies investigated the effect of miR-222-5p in cancers. As down-regulated miRNAs in GAC, miR-125-5p was identified as a tumor suppressor in glioblastoma [23], cervical cancer [24], and renal cell carcinoma [25], which was involved in proliferation, migration, and apoptosis. More researches have investigated the role of miR-145-3p in cancers, such as bladder cancer [26], lung squamous cell carcinoma [27], gallbladder cancer [28], and head and neck squamous cell carcinoma [29], which is also considered as a tumor suppressor. However, few studies have investigated the role of miRNA-379-3p; only one recent study reported that miRNA-379-5p exerted an antitumor effect by regulating tumor invasion and metastasis in hepatocellular carcinoma [30]. Unfortunately, the effect of these miRNAs on GAC has not been reported. Therefore, it is important to further reveal the mechanism and prognostic significance of these miRNAs in GAC.

Due to the highest correlation of miR-96-5p with GAC prognosis, the effect of miR-96-5p on MGC-803 cells was investigated in the present study. Consistent with previous studies [13–17], miR-96-5p silence reduced cell viability, increased cell apoptosis, and suppressed cell migration and invasion in MGC-803 cells, which suggested that miR-96-5p silence exerted tumor-promoting effect on MGC-803 cells. It is generally acknowledged that miRNAs develop biological functions by impeding translation of target mRNAs. In line with predictions, our study showed that *ZDHHC5* was identified as a target gene of miR-96-5p. ZDHHC5 is a member of the ZDHHC protein family. It encodes a DHHC type with five zinc fingers and is recognized as palmitoyl S-acyltransferase (PAT) [31]. It has been suggested that S-palmitoylation is closely associated with cancer development, and ZDHHC enzymes are the key enzymes responsible for palmitoylation [32]. Individual ZDHHC enzymes exert different effects on various cancers, either tumor suppressors or oncoproteins [32]. Previous studies have documented that high expression of ZDHHC5 is associated with the poor prognosis of glioma [33]. In addition, the report of Tian et al*.* [34] suggested that DHHC5 knockdown can dramatically inhibit cell proliferation and invasion in non–small cell lung cancer. The present study revealed that ZDHHC5 silence partly reversed the effects of miR-96-5p down-regulation on tumor cell growth and metastasis, which indicated that miR-96-5p silence inhibited tumor cell growth and metastasis by up-regulating ZDHHC5 expression. This result was inconsistent with previous studies, which may be explained that ZDHHC5 has different functions according to different cancer type [35].

In conclusion, six prognosis-related miRNAs discovered from this work include miR-96-5p, miR-125-5p, miR-145-3p, miR-222-5p, miR-379-3p, and miR- 652- 5p in GAC samples. Furthermore, down-regulated miR-96-5p markedly inhibited tumor cell growth and metastasis through targeting ZDHHC5. Current findings provide a potential molecular mechanism of miR-96-5p in GAC; however, further study is needed to investigate the mechanism and prognostic significance of these miRNAs in GAC.

## Abbreviations

Bax: BCL2 associated X, apoptosis regulator
Bcl-2: BCL2 apoptosis regulator
COX-2: cytochrome c oxidase subunit II
DEM: differently expressed microRNA
DMEM: Dulbecco’s modified Eagle’s medium
ERBB: epidermal growth factor receptor
FBS: fetal bovine serum
GAC: gastric adenocarcinoma
HE: Haematoxylin Eosin
KMsurv: R packages
miRNA: microRNA
MUT: mutant
NC: negative control
OS: overall survival
phRL-TK: phRL-TK plasmid
qPCR: quantitative polymerase chain reaction
TCGA: The Cancer Genome Atlas
WT: wild-type
ZDHHC5: zinc finger DHHC-type palmitoyltransferase 5
